The article "Use of Platelet Parameters in the Differential Diagnosis of Lung Adenocarcinoma-Associated Malignant Pleural Effusion and Tuberculous Pleural Effusion" was published in 2022. Journal: Dis Markers.

# Use of Platelet Parameters in the Differential Diagnosis of Lung Adenocarcinoma-Associated Malignant Pleural Effusion and Tuberculous Pleural Effusion

**DOI:** 10.1155/2022/5653033

**Published:** 2022-04-27

**Authors:** Ling Ai, Jingyuan Li, Ting Ye, Wenjun Wang, Yuying Li

**Affiliations:** ^1^Department of Respiratory and Critical Care Medicine, The Affiliated Hospital of Southwest Medical University, Luzhou, Sichuan 646000, China; ^2^Department of Laboratory Medicine, The Affiliated Hospital of Southwest Medical University, Luzhou, Sichuan 646000, China

## Abstract

**Background:**

Both malignant pleural effusion (MPE) and tuberculous pleural effusion (TPE) are common etiologies of pleural effusion; the present study was conducted to establish the diagnostic value of platelet parameters in the differential diagnosis of MPE and TPE.

**Methods:**

This retrospective study enrolled patients with lung adenocarcinoma-associated MPE and TPE. Platelet parameter data, including platelet count (PLT), mean platelet volume (MPV), plateletcrit (PCT), platelet distribution width (PDW), and platelet-larger cell ratio (P-LCR), were collected. Principal component analysis and multiple logistic regression modelling were carried out to assess the diagnostic value of these platelet parameters.

**Results:**

The MPE group and the TPE group enrolled 270 and 433 patients, respectively. Demographic characteristics of patients were more female and higher age in the MPE group. MPV, PDW, and P-LCR were significantly higher in MPE patients, while PLT and PCT were significantly higher in TPE patients. Principal component analysis generated two principal components (PCs) based on above platelet parameters. After adjusting for confounding factors including gender and age, multiple logistic regression showed positive association between PC1 and MPE.

**Conclusion:**

Platelet parameters were potential biomarkers in distinguishing lung adenocarcinoma-associated MPE from TPE. A patient with lower PLT and PCT and higher MPV, PDW, and P-LCR was more likely to be diagnosed as the former. Principal component analysis and multiple logistic regression performed well in improving multicollinearity, adjusting confounding factors, and identifying important risk factors for MPE.

## 1. Introduction

Pleural effusion results from an imbalance between production and absorption. It is a common complication of the body in response to systemic disorders such as cancer, infection, or inflammation [1, 2]. Both malignant pleural effusion (MPE) and tuberculous pleural effusion (TPE) are common etiologies. Most MPEs are secondary to pleural metastases of tumors from other sites, usually from lung or breast, and adenocarcinoma is the most common cell type [1–3]. TPE may be a manifestation of primary *Mycobacterium tuberculosis* (MTB) infection or related to tuberculosis reactivation [4, 5]. The management and prognosis of pleural effusion vary dramatically by etiologies. Therefore, the correct identification of MPE and TPE is important.

The article "Use of Platelet Parameters in the Differential Diagnosis of Lung Adenocarcinoma-Associated Malignant Pleural Effusion and Tuberculous Pleural Effusion" was published in 2022. Journal: Dis Markers.

The confident diagnosis of MPE is dependent on the presence of malignant cells in pleural effusion or pleural tissues. Both pleural effusion cytology and pleural biopsy pathology diagnose MPE with 100% specificity, but the sensitivity is limited to some extent [6, 7]. Some patients may also be not tolerant of thoracentesis or thoracoscopy. A series of biomarkers are shown to diagnose MPE with a little invasiveness, but the diagnostic value is still limited by many factors such as sensitivity, specificity, accessibility, and affordability [8–10].

Definitive diagnosis of TPE requires histopathological evidence of granulomatous inflammation in pleura or microbiological evidence of the organism on culture or smear [4, 5]. However, pleural biopsy is an invasive procedure [11]. Pleural effusion culture has a long time to positivity. The positive rate of acid-fast bacilli is low in pleural effusion smear [4]. Interferon-gamma release assays (IGRAs) and molecular tests of MTB are novel methods in diagnosing TPE. The former is an in vitro blood test that measures the interferon gamma released by T cells following stimulation by antigens specific to MTB. But these methods are limited by their moderate performance, high cost, and technical requirements [12].

The general platelet parameters include platelet count (PLT), mean platelet volume (MPV), plateletcrit (PCT), platelet distribution width (PDW), and platelet-larger cell ratio (P-LCR). These parameters are routinely detected in clinical practice. Changes of platelet parameters are often observed in lung cancer patients; some platelet indices are reported to be potentially diagnostic and prognostic markers of lung cancer [13–15]. The application of platelet-associated indices is also reported in the diagnosis and management of pulmonary tuberculosis [16–19]. However, the value of platelet parameters in the differential diagnosis of lung adenocarcinoma-associated MPE and TPE is still unclear. In this study, we performed principal component analysis and multiple logistic regression to characterize the association between platelet parameters and the risk of MPE.

## 2. Materials and Methods

### 2.1. Study Population

This is a retrospective study conducted in the Affiliated Hospital of Southwest Medical University from July 2013 to May 2021. The diagnoses of malignant pleural effusion (MPE) and tuberculous pleural effusion (TPE) were made according to corresponding diagnostic criteria. Data of platelet count (PLT), mean platelet volume (MPV), plateletcrit (PCT), platelet distribution width (PDW), and platelet-larger cell ratio (P-LCR) were collected in these patients. The study protocol was approved by the ethics committee of the Affiliated Hospital of Southwest Medical University.

The article "Use of Platelet Parameters in the Differential Diagnosis of Lung Adenocarcinoma-Associated Malignant Pleural Effusion and Tuberculous Pleural Effusion" was published in 2022. Journal: Dis Markers.

### 2.2. Inclusion and Diagnostic Criteria of Participants

The pleural effusion would be diagnosed as MPE when pleural effusion cytology or pleural biopsy pathology was positive for malignant cells. MPE would be classified as lung adenocarcinoma associated when the malignant cell was judged as adenocarcinoma cell according to morphological features, and the primary tumor site was judged as lung according to immunohistochemical evidences or radiological evaluation. The patient would be excluded when (1) the pleural effusion was not MPE or not lung adenocarcinoma associated; (2) antineoplastic treatments, including chemotherapy, radiotherapy, immunotherapy, and targeted therapy, were received before MPE was diagnosed in our hospital; (3) data of platelet parameters were missed.

The pleural effusion would be diagnosed as TPE when (1) positive mycobacterial culture, acid-fast staining, or polymerase chain reaction (PCR) in pleural effusion or pleural biopsy tissues, and (2) granuloma in pleural biopsy, with or without caseous necrosis, in the absence of other causes of granulomatous lung disease. Patients with missed data of platelet parameters were excluded.

### 2.3. Sample Acquisition, Preparation, and Laboratory Analysis

Pleural biopsy was conducted by experienced doctors through medical thoracoscopy. Lateral decubitus position was taken in the patient postartificially induced pneumothorax. A semirigid thoracoscope was inserted into the pleural space postlocal infiltration anesthesia and thoracotomy. Biopsy was then performed in abnormal sites of the parietal pleura under direct visualization of the pleural space. The pleural biopsy tissues were stored in formaldehyde and sent for pathological diagnosis.

In pleural effusion cytology, thoracentesis was conducted in patient directed by the ultrasound. Approximately 100 ml pleural effusion was collected in the sterile container and centrifuged at 1500 rpm for 15 min at room temperature. The liquid supernatant was removed, and the pellet was recollected and resuspended. Then, smears were prepared from ThinPrp®2000 (Hologic Inc., USA), stained with hematoxylin-eosin staining, and sent for cytological diagnosis.

For platelet parameter test, approximately 3-4 ml venous blood sample was collected in an EDTA-K2 anticoagulant tube on admission. Platelet parameters, including PLT, MPV, PCT, PDW, and P-LCR, were measured using Maccura (XN-9000, China) according to the manufacturer's protocols.

The article "Use of Platelet Parameters in the Differential Diagnosis of Lung Adenocarcinoma-Associated Malignant Pleural Effusion and Tuberculous Pleural Effusion" was published in 2022. Journal: Dis Markers.

### 2.4. Statistical Analysis

The normality of all quantitative data was tested by the Kolmogorov–Smirnov test. Normally distributed data were presented as mean ± standard deviation (SD); comparisons between groups were carried out using Student's *t*-test. Nonnormally distributed data were presented as median and interquartile range; comparisons between groups were carried out using the Mann–Whitney *U* test. Qualitative data was analyzed through chi-square test. Principal component analysis was carried out to determine and solve the multicollinearity between platelet parameters. Multiple logistic regression was carried out to screen clinically significant eigenvalues and identify confounding factors. All statistical analyses were performed using GraphPad Prism 9.0.2 Software (San Diego, CA, USA). *P* < 0.05 was considered to be statistically significant.

## 3. Results

### 3.1. General Characteristics of Enrolled Participants

The present study retrospectively enrolled patients with lung adenocarcinoma-associated MPE and TPE in the Affiliated Hospital of Southwest Medical University between July 2013 and May 2021. A total of 382 patients were initially diagnosed as MPE, of whom 102 were excluded for nonlung adenocarcinoma-associated or previous antineoplastic treatments, and 10 patients were excluded for missed data of platelet parameters. Finally, 270 eligible patients were enrolled in the MPE group. The diagnosis of lung adenocarcinoma-associated MPE was evidenced by pleural effusion cytology in 188 patients, which was evidenced by pleural biopsy in 31 patients. Other 51 patients were supported by both pleural effusion cytology and pleural biopsy pathology. In the TPE group, 433 eligible patients were enrolled postexclusion of 20 patients for missing data. All of the 433 patients were positive for granulomatous inflammation in parietal pleura, of whom 90 and 66 patients were also positive for TB-DNA detected by PCR and caseous necrosis in pleural tissues, respectively.

As it was listed in Table 1, the present study included two groups: lung adenocarcinoma-associated MPE group (*n* = 270, including 143 male and 127 female) and TPE group (*n* = 433, including 296 male and 137 female). Both the age and gender composition were significantly different between two groups, with higher age and proportion of female patients in the MPE group (*P* < 0.0001). In platelet parameters, no data satisfied the normal distribution. MPV, PDW, and P-LCR in the MPE group were significantly higher than those in the TPE group (*P* < 0.0001), while PLT and PCT showed significantly higher values in the TPE group (*P* < 0.0001).

The article "Use of Platelet Parameters in the Differential Diagnosis of Lung Adenocarcinoma-Associated Malignant Pleural Effusion and Tuberculous Pleural Effusion" was published in 2022. Journal: Dis Markers.

### 3.2. Principal Component Analysis of Platelet Parameters

All platelet parameters showed significant differences between lung adenocarcinoma-associated MPE group and TPE group, with higher MPV, PDW, and P-LCR in the former and higher PLT and PCT in the latter. Principal component analysis (PCA) was therefore carried out to estimate and eliminate the multicollinearity between above variables. Principal components (PCs) were selected based on parallel analysis.

The model generated five PCs; corresponding eigenvalue in PC1 to PC5 was 2.731, 1.408, 0.776, 0.069, and 0.015, respectively. PC1 together with PC2 explained cumulative 82.79% of the variation within the dataset (Figure 1(a)). Therefore, PC scores of PC1 and PC2 were then selected for further logistic analysis. Based on distribution features of plots in PC scores, capacity seems to be comparable between PC1 and PC2 in distinguishing MPE from TPE (Figure 1(b)). Eigenvectors and component loadings of PC1 and PC2 were listed in Table 2. Except for the low absolute value of 0.018 between PC2 and PDW, absolute values of eigenvectors between PCs and other variables were comparable. Accordingly, PC1 was characterized by PLT, MPV, PCT, PDW, and P-LCR, while PC2 was mainly characterized by PLT, MPV, PCT, and P-LCR. Positive component loadings were obtained between PLT as well as PCT and PC1; this means that PC1 may increase when PLT or PCT increased. Negative component loadings between other variables and PCs showed negative correlations between them. The absolute value of loading was just 0.022 between PC2 and PDW; this further evidenced the aforementioned poor coefficient of PDW. Besides, eigenvector between MPV and PCs was comparable to that between P-LCR and PCs; component loading between MPV and PCs was also comparable to that between P-LCR and PCs; this showed possibly strong multicollinearity between MPV and P-LCR (Figure 1(c) and Table 2).

### 3.3. Multiple Logistic Regression of PCs and Demographic Data

Multicollinearity of platelet parameters was shown in principal component analysis and then PCs were produced. Consequently, PCs instead of initial platelet parameters were included in variables of the multiple logistic regression. Demographic data of gender and age were also included in the modelling to adjust to potential confounding factors. Positive and negative outcome of *Y* was, respectively, represented by lung adenocarcinoma-associated MPE and TPE. Gender, age, PC1, and PC2 was then set as *X*1, *X*2, *X*3, and *X*4, respectively. According to the logistic regression modelling, variance inflation factor (VIF) was 1.019, 1.072, 1.068, and 1.023, respectively, in *X*1 to *X*4. After adjusting for potential confounding factors of gender and age, positive association was showed between PC1 and risk of MPE with an odds ratio of 1.292 (*P* < 0.0001), while no significant association was found between PC2 and MPE (*P* > 0.05, Table 3). With a classification cutoff value of 0.5, the positive and negative predictive power of this model was 78.1% and 68.1%, respectively (Figure 2(a)). An ROC (receiver operating characteristic) curve was also generated in the logistic regression modelling, and an AUC (area under the curve) of 0.8235 was obtained (Figure 2(b)). Akaike's corrected information criterion (AICc) of 704.3 and 938.4 was, respectively, calculated in selected model and intercept-only model; this means that the selected model fit the included data. The Hosmer-Lemeshow test also showed that this model was fit (*P* > 0.05).

The article "Use of Platelet Parameters in the Differential Diagnosis of Lung Adenocarcinoma-Associated Malignant Pleural Effusion and Tuberculous Pleural Effusion" was published in 2022. Journal: Dis Markers.

## 4. Discussion

In the present study, significantly higher MPV, PDW, and P-LCR while lower PLT and PCT were observed in lung adenocarcinoma-associated MPE patients. The MPE group also had significantly higher age and proportion of female patients than the TPE group. The two PCs generated by principal component analysis contributed to 82.79% of the total variance of all platelet variables. After adjusting for potential confounding factors including age and gender, multiple logistic regression showed positive association between PC1 and MPE. Accordingly, increased MPV, PDW, and P-LCR and decreased PLT and PCT correlated with higher suspicious of lung adenocarcinoma-associated MPE.

Pleural effusion is the pathological accumulation of fluid in pleural space. Both MPE and TPE are common etiologies of it and generally lead to exudate, but their treatment strategies and prognoses are quite different [20]. Lung adenocarcinoma is responsible for most MPEs [2, 3]. Accurate etiological diagnosis is essential for further management. Pleural effusion cytology and pleural biopsy pathology help to determine malignant cell types and molecular genetic profiles of MPE. But the diagnostic sensitivity of cytology is limited and varies with underlying cancer types [6, 7, 21]. Pleural biopsy has higher sensitivity, but it is limited by cost, invasiveness, and expertise availability [6]. Many noninvasive biomarkers including tumor markers are also reported in diagnosing MPE. However, the accuracy is insufficient to confirm MPE when these biomarkers are used either alone or in combination [8, 9, 22].

The confident diagnosis of TPE is based on microbiological or histopathological evidences of MTB infection [23, 24]. But smear and culture of MTB from pleural effusion are, respectively, limited by low positive rate and long time to positivity. Pleural biopsy is requisite to make histopathological diagnosis, but it is an invasive procedure and unavailable in many hospitals as described above [23]. Novel methods such as molecular tests are limited by affordability, accessibility, and diagnostic performance [24]. The differential diagnosis of MPE and TPE is therefore still a challenging problem. Traditional diagnostic approaches need improvement and optimization.

The article "Use of Platelet Parameters in the Differential Diagnosis of Lung Adenocarcinoma-Associated Malignant Pleural Effusion and Tuberculous Pleural Effusion" was published in 2022. Journal: Dis Markers.

Platelet plays important roles in the regulation of hemostasis and thrombus formation. It also regulates inflammation, innate immunity, antimicrobial host defense, atherogenesis pathogenesis, tumor growth, and metastasis [25–27]. Platelet parameters including PLT, MPV, PCT, PDW, and P-LCR can be easily obtained from routine laboratory work. These platelet parameters are demonstrated to help diagnosing a series of vascular, inflammatory, metabolic, and malignant diseases [28–31]. The interaction of tumor cells and platelets is a prerequisite for successful hematogenous metastatic dissemination. Significantly higher PLT, MPV, PCT, and PDW have been reported in lung cancer patients when compared with healthy controls [32–34]. Elevated PLT was also associated with higher risk of pleural metastasis and poorer prognosis of lung cancer patients [35, 36]. This revealed potentially diagnostic and prognostic value of these platelet parameters in lung cancer. In terms of MTB infection, pulmonary tuberculosis patients were reported to have significantly higher PLT, MPV, PCT, and PDW than healthy controls or other benign lung diseases patients [19, 37]. Above platelet parameters are therefore also possibly diagnostic biomarkers of pulmonary tuberculosis.

However, data of these platelet parameters in pleural effusion patients with different etiologies is unavailable in most reported studies. Their diagnostic value in distinguishing MPE from TPE remains unclear. In the present study, we verified the hypothesis that platelet parameters are potential biomarkers in the differential diagnosis of lung adenocarcinoma-associated MPE and TPE. The results revealed significant differences of all platelet parameters between two groups and accordingly indicated their diagnostic value. Principal component analysis together with multiple logistic regression helped to identify and adjust the impact of confounding factors and multicollinearity between parameters. The model produced in the regression concluded that all platelet parameters are potentially diagnostic biomarkers. Patients with higher MPV, PDW, and P-LCR and lower PLT and PCT are more likely to be diagnosed as lung adenocarcinoma-associated MPE rather than TPE. MPV and P-LCR have strong multicollinearity and comparable diagnostic value; this may be explained by the fact that both MPV and P-LCR are indexes reflecting the size of platelet [38].

The article "Use of Platelet Parameters in the Differential Diagnosis of Lung Adenocarcinoma-Associated Malignant Pleural Effusion and Tuberculous Pleural Effusion" was published in 2022. Journal: Dis Markers.

The present study has some limitations. First, this was a retrospective study of patients with MPE and TPE, and possibility of some bias could not be completely excluded. Second, the study population was enrolled from a single center with limited cohort size, so it could not fully represent populations from other regions and countries. Third, prognostic data such as overall survival of these patients was unavailable. A multicenter prospective study that enrolled more participants is therefore warranted to further confirm these results and clarify corresponding mechanisms.

## 5. Conclusions

In summary, the present study revealed for the first time that platelet parameters are promising biomarkers for the differential diagnosis of lung adenocarcinoma-associated MPE and TPE. Lung adenocarcinoma-associated MPE patients tend to have higher MPV, PDW, and P-LCR but lower PLT and PCT than TPE patients. The diagnostic value of PLT, MPV, and P-LCR is superior to that of PCT and PDW.

## Figures and Tables

**Figure 1:** Principal component analysis of platelet variables. (a) Proportion of variance plot of PCs. (b) Score plot of PCs with symbol fill color of diagnosis. (c) Loading plot of PCs.

**Figure 2:** Multiple logistic regression of PCs postadjustments of confounding factors. (a) Predicted vs. observed graph of the logistic regression modelling. (b) ROC curve of the logistic regression modelling.

**Table 1:** Comparison of clinical features and platelet parameters between two groups.

Variable	MPE group	TPE group	*P* value
Number of patients	270	433	
Gender (male/female)	143/127	296/137	<0.0001
Age (years)	65 (54-73)	45 (28-59)	<0.0001
PLT (×10^9^/l)	279.0 (221.8-335.3)	325.0 (266.0-392.5)	<0.0001
MPV (fl)	10.1 (9.275-11.0)	9.6 (8.75-10.5)	<0.0001
PCT	0.28 (0.23-0.33)	0.31 (0.26-0.37)	<0.0001
PDW (%)	15.75 (12.38-16.3)	15.3 (10.85-16)	<0.0001
P-LCR (%)	26.45 (20.85-33.65)	22.2 (16.9-28.9)	<0.0001

Quantitative data were presented as medians (25th to 75th percentiles).

**Table 2:** Eigenvectors and component loadings of PCs.

	PC1	PC2
Eigenvectors		
PLT	0.518	-0.398
MPV	-0.480	-0.462
PCT	0.381	-0.646
PDW	-0.342	-0.018
P-LCR	-0.490	-0.458
Component loadings		
PLT	0.856	-0.472
MPV	-0.793	-0.548
PCT	0.63	-0.767
PDW	-0.565	-0.022
P-LCR	-0.809	-0.544

**Table 3:** Results of multiple logistic regression analysis.

	Odds ratios	95% confidence interval	*P* value
Gender (male)	2.383	1.629-3.511	<0.0001
Age	0.929	0.916-0.941	<0.0001
PC1	1.292	1.152-1.454	<0.0001
PC2	0.928	0.796-1.081	0.3397

The article "Use of Platelet Parameters in the Differential Diagnosis of Lung Adenocarcinoma-Associated Malignant Pleural Effusion and Tuberculous Pleural Effusion" was published in 2022. Journal: Dis Markers.

## Data Availability

The raw data required to reproduce these findings cannot be shared at this time as the data also forms part of an ongoing study.
